This article has been retracted.

# The Use of Tooth Particles as a Biomaterial in Post-Extraction Sockets. Experimental Study in Dogs

**DOI:** 10.3390/dj6020012

**Published:** 2018-05-06

**Authors:** José Luis Calvo-Guirado, José Eduardo Maté-Sánchez de Val, María Luisa Ramos-Oltra, Carlos Pérez-Albacete Martínez, María Piedad Ramírez-Fernández, Manuel Maiquez-Gosálvez, Sergio A Gehrke, Manuel Fernández-Domínguez, Georgios E. Romanos, Rafael Arcesio Delgado-Ruiz

**Affiliations:** 1 Faculty of Health Sciences, Universidad Católica de Murcia (UCAM), Campus de los Jerónimos N° 135, Guadalupe, 30107 Murcia, Spain; jemate@ucam.edu (J.E.M.-S.d.V.); mlramos@ucam.edu (M.L.R.-O.); cperezalbacete@ucam.edu (C.P.-A.M.); 2 Department of Epidemiology, Universidad Católica de Murcia (UCAM), 30107 Murcia, Spain; mpramirez@ucam.edu; 3 Faculty of Health Sciences, Department of Oral and Implant Dentistry Universidad Católica de Murcia (UCAM), 30107 Murcia, Spain; sergio.gehrke@hotmail.com; 4 Biotecnos Research Center—Tecnología e Ciencia Ltd., 11100 Montevideo, Uruguay; sergio.gehrke@hotmail.com; 5 Faculty of Dentistry, Department of Oral and Implant Dentistry, San Pablo University CEU, Group HM (Hospital Madrid), 28050 Madrid, Spain; clinferfun@yahoo.es; 6 Department of Periodontology, School of Dental Medicine, Stony Brook University, New York, 11794 NY, USA; Georgios.Romanos@stonybrookmedicine.edu; 7 Department of Prosthodontics and Digital Technology, School of Dental Medicine, Stony Brook University, New York, 11794 NY, USA; Rafael.Delgado-Ruiz@stonybrookmedicine.edu

**Keywords:** Smart Dentin Grinder, tooth particles, autogenous particulate tooth graft, socket preservation, dog study

## Abstract

**Objectives**: The objective of this study was to evaluate new bone formation derived from freshly crushed extracted teeth, grafted immediately in post-extraction sites in an animal model, compared with sites without graft filling, evaluated at 30 and 90 days. **Material and Methods**: The bilateral premolars P2, P3, P4 and the first mandibular molar were extracted atraumatically from six Beagle dogs. The clean, dry teeth were ground immediately using the Smart Dentin Grinder. The tooth particles obtained were subsequently sieved through a special sorting filter into two compartments; the upper container isolating particles over 1200 μm, the lower container isolated particles over 300 μm. The crushed teeth were grafted into the post-extraction sockets at P3, P4 and M1 (test group) (larger and smaller post-extraction alveoli), while P2 sites were left unfilled and acted as a control group. Tissue healing and bone formation were evaluated by histological and histomorphometric analysis after 30 and 90 days. **Results**: At 30 days, test site bone formation was greater in the test group than the control group (*p* < 0.05); less immature bone was observed in the test group (25.71%) than the control group (55.98%). At 90 days, significant differences in bone formation were found with more in the test group than the control group. No significant differences were found in new bone formation when comparing the small and large alveoli post-extraction sites. **Conclusions**: Tooth particles extracted from dog’s teeth, grafted immediately after extractions can be considered a suitable biomaterial for socket preservation.

## 1. Introduction

There is compelling evidence that immediate grafting of extraction sockets using various ridge preservation techniques—including the placement of graft materials and/or the use of occlusive membranes—will prevent alveolar bone loss during the repair phase of wound healing. However, the technique lacks the capacity to promote osteogenesis and osteoinduction, and so its usefulness is limited in terms of the formation of viable bone [1].

Human demineralized dentin matrix created from extracted human teeth was first developed in 2008 and its use in implant dentistry has been evaluated on the basis of its osteoinductive, osteoconductive, and remodeling capacity. By weight, dentin and bone are composed of 30% collagen, 60% hydroxyapatite, and 10% body fluid [2,3,4,5]; by volume, they are composed of 10% liquid, 20% collagen, and 70% hydroxyapatite. These proportions place bone and dentin in the same class of material as biomaterials that consist of collagen and ceramic material [6,7,8,9,10].

Kim and his team have been investigating the development of biomaterials using human teeth since 1993, and have recently reported the promising results of their research [11,12,13,14,15,16,17]. Tooth dentin and cementum structure are similar to membranous bone in their mineral and protein composition; when new bone matrix is directly deposited on membranous surfaces, this results in ankylosed dentin-bone interfaces [18,19]. When avulsed teeth are re-implanted back into their sockets or when extracted teeth are processed immediately after being extracted into a particulate dentin graft that is inserted into freshly extracted socket in the same patient, this also creates ankylosed interfaces [20,21,22].

The “Smart Dentin Grinder”^TM^ device has been designed to crush and sort extracted teeth into tooth particles of specific sizes. A chemical cleanser and a buffer are applied for 15–20 mins to eliminate bacteria. This novel procedure can be indicated for most tooth extractions, although endodontically treated teeth are counter-indicated due to contamination by foreign materials.

The objective of this study was to evaluate immature bone and new bone formation after filling fresh extraction sockets in an animal model with tooth particle graft compared with empty sockets, after a 90-day follow-up.

## 2. Material and Methods

Six Beagle dogs about one year old, weighing 14–15 kg each were used in the study. The University of Murcia Ethics Committee for Animal Research approved the study protocol A1320140404 (12-02-2015), which followed guidelines established by the Directive of the Council of the European Union of February 1, 2013/53/CEE, guidelines for animal studies.

The animals were quarantined for the application of rabies and vitamin vaccines. The animals were kept in cages before and after the operation and received appropriate veterinary attention during the study period. All the animals presented intact dental arches, without viral or fungal mouth lesions.

The animals were pre-anesthetized with 10% zolazepam at 0.10 mL/kg and acepromazine maleate (Calmo-Neosan®, Pfizer, Madrid, Spain) 0.12–0.25 mg/kg and medetomidine 35 mg/kg (Medetor 1 mg, Virbac, CP-Pharma Hand-elsgesellschaft GmbH, Burgdorf, Germany). The mixture was injected intramuscularly into the quadriceps femoris. The animals were taken to the operating theatre where, at the first opportunity, an intravenous catheter (diameter 22 G or 20 G) was inserted into the cephalic vein, and propofol infusion was administered at a rate of 0.4 mg/kg/min at a constant infusion rate.

Anesthetic maintenance was performed with volatile anesthetics and the animals underwent tracheal intubation with a Magill probe for the adaptation of the anesthetic device and for the administration of volatile isoflurane diluted in oxygen (2 V%). In addition, local anesthesia (Articaine 40 mg, 1% epinephrine, Normon®, Madrid, Spain) was administered at the surgical sites. These procedures were carried out under the supervision of a veterinary surgeon.

Mandibular premolars and first molars (P2, P3, P4, M1) were extracted bilaterally (Figure 1) under general anesthesia.

Teeth with multiple roots were hemisectioned in bucco-lingual direction, protecting the remaining bony walls. Immediately after extraction, the clinician eliminated the organic coating of the root surfaces that includes periodontal ligament tissue and bacterial biofilm, which was removed using a tungsten carbide bur, or hand-piece drill and water.

The teeth were cleaned, dried with an airflow syringe, and crushed immediately after extraction isolating the crown and root using the “Smart Dentin Grinder” (Bioner Sistemas Implantológicos, Barcelona, Spain), specially designed for this procedure. The tooth particles obtained were sized at 300–1200 μm, which were sieved through a special sorting system into two compartments: the upper container has a grid to isolate larger particles of over 1200 μm, while the lower container is more rigid, allowing the accumulation of smaller particles of over 300 μm (Figure 2).

More than 95% of the tooth particulate accumulates in a sterile “drawer chamber” that isolates particles of 300–1200 μm (the optimal size for achieving an osteogenic interaction at the grafted site), isolating smaller and larger particles in separate trays. The particulate volume is about 2–3 times greater than the original volume of the tooth. The particle size criteria is based on the fact that small particles facilitate quick bone resorption (300 μm) and bone maintenance, while larger particles (over 1200 μm) protect against and reduce bone resorption. Both type of tooth particles were obtained in two different compartments and the proportion of both particles used were 80% of big particles and 20% of small particles to avoid inflammation.

The particulate teeth were immersed in a basic alcohol cleanser in a sterile container for 15 min to dissolve all organic waste and bacteria. The particles were then washed with sterile saline for 5 min. Then the particles were dried, and the small and large tooth particles were mixed. The particulate was then grafted into post-extraction sites of premolars P3, P4 and first molar M1 (test group), they were filled with freshly extracted teeth (Figure 3), while the premolar P2 sockets on both sides remained unfilled, acting as control sites.

Ethanol 70% denatures and precipitates proteins and so is bactericidal. The present experiment used a 30% solution of 70% ethanol, which, in addition to its main bactericidal action, strongly enhances the action of NaOH, which eliminates organic compounds, while ethanol does not. So, the combination of ethanol and NaOH completely dissolves every organic substance and acts as a very effective disinfectant. Ethanol only affects organic compounds on the outside surface of the mineral (external organic substances). It does not penetrate the mineral and so does not affect collagen trapped in the mineral itself (which, in any case, is not infected).

Continuous non-absorbable sutures (Silk 3.0, Lorca Marin, Lorca, Murcia, Spain) were used to protect and maintain the grafted areas (Figure 4). The stitches were removed after 15 days.

Mandibular teeth from canine to canine were maintained and no surgeries were performed in the upper maxilla. All surgical techniques were performed under the supervision of the University veterinarian, assigned to the University of Murcia’s Animal Research Unit.

During the surgical procedure, the animals were hydrated with glucose-saline (250 cm^3^) to aid post-surgical recovery. Following the guidelines established by the animal research ethics committees, anti-inflammatory and antibiotic drugs were administered after surgery and every other day for seven days to prevent postoperative infection and inflammation: the anti-inflammatory, Metacam® (Boehringer, Ingelheim Vetmedica, Ingelheim, Germany), 1–2 mL intramuscularly; and the antibiotic Alsir® (enrofloxacin), 2 mL intramuscularly.

After surgery, the dogs were transferred to individual cages where they remained under veterinary supervision. The animals were fed ad-libitum with a soft diet during the study period.

The animals’ soft tissues were disinfected and cleaned with a mouthwash based on seawater: Sea 4 Encías (Blue Sea Laboratories, Alicante, Spain).

After 30 and 90 days healing, a local anesthetic was applied to the buccal and lingual gums and crestal incisions were made in the area regenerated from the canine to the second molar (Figure 5). A full thickness mucoperiosteal flap was lifted and, using a 3 mm diameter trephine bur, biopsies were extracted from the control sites and from the areas of regenerated bone on both sides of the mandible (Figure 6).

### 2.1. Histology

The bone cores obtained were individually preserved in 10% formaldehyde for 20 days. The samples were then decalcified for 30 days using TBD-2 (Anatomical Pathology International, Runcorn, Cheshire, UK). After dehydration and inclusion in paraffin, sections of 20 μm thickness were prepared; samples were stained with picrosirius-hematoxylin and hematoxylin to distinguish between immature and mature bone.

For histomorphometric analysis, images were enlarged 20×, and eight fields per sample were evaluated digitally (using a DP12 digital camera, Olympus, Nagano, Japan). Microimage 4.0 software (Media Cybernetics, Silver Spring, MD, USA) was used for image analysis.

All analyses were carried out by the same technician, who was blinded to each sample’s group assignation (test or control).

The total area of newly formed bone and connective tissue were evaluated and the percentage of immature bone was measured.

### 2.2. Statistical Analysis

Statistical analysis was performed using SPSS 21.0 software (SPSS, Chicago, IL, USA). Descriptive statistics were calculated (mean and standard deviation) for both groups. For the comparison of means, a non-parametric Friedman test was applied with a significance level of 95% (*p* < 0.05). The Mann–Whitney U test, a non-parametric test, was applied and the ANOVA test was used to analyze the differences between variables.

## 3. Results

Sample sizes were 3.5 mm in diameter by 8.5 mm in length (6 alveolus per dog) and 6 mm by 10 mm length (2 alveolus per dog) a total of 36 small and 12 big alveolus filled for both test and control specimens.

### 3.1. Histological Analysis at 30 Days

Control samples showed large amounts of newly formed immature bone covering the bone defect, and highly disorganized tissues with high rates of cellularity and large medullary cavities.

The tooth particulate group showed newly formed bone with irregular disposition and high levels of capillarity, but to a lesser extent than the control group (Figure 7a,b).

### 3.2. Histomorphometric Evaluation

At 30 days, new bone formation was 72.35 ± 0.98% in the defects treated with tooth particle grafts (test group), while in the untreated defects (control group) new bone formation was 55.87 ± 0.32%, with statistically significant difference between the groups (*p* < 0.05) (Table 1).

At 90 days, new bone was 77.18 ± 0.76% in defects treated with tooth particle grafts (test group), compared with the control group (58.92 ± 0.32%) with statistically significant difference (*p* < 0.05)*. (Table 2).

### 3.3. Histological Analysis at 90 Days

The control group showed greater bone organization compared with the 30-day evaluation. All bone defects were completely covered by newly formed osteons, while other areas were occupied by non-organized immature bone (Figure 7c). The test group showed mature newly formed bone, well organized by multiple osteons throughout the entire bone (Figure 7d).

### 3.4. Histomorphometric Evaluation of Immature Bone

At 30 days, histomorphometric analysis found immature bone (25.71 ± 0.25%) in defects treated with tooth particulate with significant difference between the test and control groups (55.98 ± 0.16%). At 90 days, histomorphometric analysis found total immature bone of 14.2 ± 0.66% in the test group with significant differences in comparison with the control group (35.17 ± 0.74%) (Table 3).

## 4. Discussion

Our last published work described how fresh extraction sockets can be grafted with tooth particles made by crushing the extracted teeth; bone formation was evaluated after 30 days and 90 days (the early stages of healing) finding more immature and mature bone at test sites than control sites at both study times 22). Although in the present study, the statistical method was different, the present results were similar to the earlier study, observing more immature bone at 30 days and more mature bone at 90 days, with less connective tissue. These data show how the tooth particles resorb and are replaced by new bone at 90 days.

Teeth that suffer trauma have ankylosed roots, which continuously resorb over time and are replaced by bone, eventually resorbing the entire root, while the alveolar bone is conserved during this period. Malmgren et al. described the decoronation method, offering possible explanations for the favorable outcome of this technique and proposing guidelines for deciding the correct time for intervention. After decoronation, the alveolar ridge was maintained in buccal/palatal direction, and the bone level increased, so maintaining normal alveolar conditions [23]. Pang et al. used autogenous demineralized dentin matrix from extracted teeth to graft extraction sockets and augment the vertical dimension; this was found to be as effective as augmentation using an organic bovine bone [24].

The present results reveal a close and direct interaction between mineralized dentin, bone matrix, and the grafted tooth particle material. When the extraction of a tooth is necessary, the Smart Dentin Grinder makes it possible to prepare the tooth particles from the freshly extracted autologous tooth, ready for use in as little as 15 min during a single surgical session. With no antigenicity, it improves bone remodeling capabilities and can be considered a viable graft option given its autogenous origin and favorable clinical and histological results. Moreover, despite its inductive properties, mineralized dentin integrates into newly formed bone, creating a stable site for dental implant insertion. In fact, several clinical studies have shown that implant insertion and loading can be performed in both upper and lower jaws as early as 2–4 months after grafting with crushed and demineralized tooth and bone [25,26].

Since mineralized dentin is remodeled very slowly, as compared with cortical bone, the aesthetic and structural integrity of the alveolar ridge is maintained for many years [27,28]. The patient’s tooth is comparable to autogenous bone graft material and possesses all the properties of the patient´s bone due to its very similar components to bone, making it very useful in many clinical situations. The teeth and the jaw have a high level of affinity, with similar physical, chemical structures and composition [24].Kim et al. reported that 90% of the organic component of the tooth are type I collagen, which is very important in bone calcification [27,28,29,30,31,32]. 

Autogenous demineralized dentin matrix from extracted tooth grafted to extraction sockets for the augmentation of vertical dimension was as effective as augmentation using anorganic bovine bone. Both groups showed favorable wound healing, similar amount of implant stability, and histologically confirmed new bone formation. Thus, the results of this study suggest that autogenous tooth graft material is a viable option for alveolar bone augmentation following dental extraction [33].

It also overcomes patients’ rejection of materials derived from animal or synthetic sources, as well as providing excellent biocompatibility without provoking an immune response, foreign material reaction, or infection. Unless it is contaminated by an infectious lesion, a tooth does not cause problems, even when the root tip is left in the alveolar bone. The use of the patient’s own tooth is entirely legal, providing the patient agrees. 

In the present study, the crushed tooth particulate produced more bone regeneration at 90 days than control samples. As the dentin graft maintains the collagen structure, it preserves both the height and width of bone crests.

## 5. Conclusions

Within the limitations of the present animal study, it would appear that tooth particle graft (both enamel and dentin) can be viewed as a useful autogenous biomaterial for socket preservation due to its similar characteristics to autologous bone. Currently, this graft material can be used in combination with autologous bone debris as an excellent graft material without compromising the capacity for bone regeneration.

## Figures and Tables

**Figure 1:** (**a**) Bilateral mandibular premolars P2, P3, P4 and first molar to be extracted; (**b**) Post-extraction sockets of mandibular premolars and first molars.

**Figure 2:** (**a**) Smart dentin grinder device; (**b**) Dog’s extracted premolar teeth inside grinding chamber; (**c**) Tooth particles of 300–1200 microns obtained after using the grinding device.

**Figure 3:** Ground tooth particles filling P3, P4 and first Molar M1 sockets. No material was placed into premolar P2 sockets, which acted as control sites.

**Figure 4:** Continuous non-absorbable sutures (Silk 3.0, Lorca Marin, Lorca, Murcia, Spain) were used to protect and maintain the grafted areas.

**Figure 5:** Healing bone in regenerated area at 90 days.

**Figure 6:** Core sites of tooth particles and control sites at 90 days.

**Figure 7:** (**a**) Control group showed large quantity of newly formed immature formed bone covering the bone defect; (**b**) tooth particle group samples were characterized by the presence of newly formed bone of irregular disposition, with high levels of cellularity (test group); (**c**) images show newly formed osteons with non-organized immature bone in the control group at 90 days; (**d**) tooth particle group (test group) showing newly formed well organized mature bone at 90 days.

**Table 1:** Mean values ± standard deviation of new bone and connective tissue quantity at 30 days statistically significant difference (*p* < 0.05)*.

Evaluation at 30 Days	Tooth Particulate Mean ± SD % Test Group	Control Group	*p*-Value
New bone	72.35 ± 0.98 *	55.87 ± 0.32	<0.011 *
Connective tissue	22.82 ± 0.54	31.76 ± 0.61	<0.791

* statistically significant difference (*p* < 0.05).

**Table 2:** Mean values ± standard deviation of new bone formation and connective tissue at 90 days (*p* < 0.05).

Evaluation at 90 Days	Tooth Particulate Mean ± SD %	Control	*p*-Value
New bone	77.18 ± 0.76	59.92 ± 0.32	<0.017 *
Connective tissue	10.68 ± 0.42	22.89 ± 0.27	<0.561

* statistically significant difference (*p* < 0.05).

**Table 3:** Mean values ± standard deviation of the quantity of immature bone quantity at 30 and 90 days (*p* < 0.05)*.

	Quantity OF Immature Bone	
	Tooth Particulate (%) Mean ± SD Test Group	Control (%) Mean ± SD Control Group
30 days	25.71 ± 0.25 *	55.98 ± 0.16
90 days	14.2 ± 0.66 *	35.17 ± 0.74

* statistically significant difference (*p* < 0.05).
